The article "Association between the UGT1A1*28 allele and hyperbilirubinemia in HIV-positive patients receiving atazanavir: a meta-analysis" was published in 2019. Journal: Biosci Rep.

# Association between the UGT1A1*28 allele and hyperbilirubinemia in HIV-positive patients receiving atazanavir: a meta-analysis

**DOI:** 10.1042/BSR20182105

**Published:** 2019-05-02

**Authors:** Pengqiang Du, Aifeng Wang, Yongcheng Ma, Xingang Li

**Affiliations:** 1 Department of Pharmacy, Fuwai Central China Cardiovascular Hospital, Zhengzhou 450046, China; 2 Department of Pharmacy, Beijing Friendship Hospital, Capital Medical University, Beijing 100050, China

**Keywords:** UGT1A1*28, atazanavir, hyperbilirubinemia, meta analysis

## Abstract

**Objectives** The uridine diphosphate glucuronosyltransferase 1A1 (UGT1A1)*28 allele in HIV-positive patients receiving atazanavir (ATV) might be associated with the risk of hyperbilirubinemia. Owing to mixed and inconclusive results, a meta-analysis was conducted to systematically summarize and clarify this association.

**Methods** Based on a comprehensive search of PubMed, Embase and Web of Science databases, studies investigating the association between UGT1A1 alleles and hyperbilirubinemia was retrieved. We evaluated the strength of this relationship using odds ratios (ORs) with 95% confidence intervals (CIs). Sensitivity analysis was performed by removing each study one at a time and calculating the pooled ORs of the remaining studies to test the robustness of the meta-analysis results. The Q statistic and the *I^2^* index statistic were used to assess heterogeneity. Publication bias was evaluated using Orwin’s fail-safe N test.

**Results** A total of six individual studies were included in this meta-analysis. A significantly increased risk of hyperbilirubinemia was observed in HIV-positive patients receiving ATV with the UGT1A1*1/*28 or UGT1A1*28/*28 genotype, and the risk was higher with the UGT1A1*28/*28 genotype than with the UGT1A1*1/*28 genotype. (UGT1A1*28/*28 versus UGT1A1*1/*28: OR = 3.69, 95%CI = 1.82–7.49; UGT1A1*1/*28 versus UGT1A1*1/*1: OR = 3.50, 95%CI = 1.35–9.08; UGT1A1*28/*28 versus UGT1A1*1/*1: OR = 10.07, 95%CI = 4.39–23.10). All of the pooled ORs were not significantly affected by the remaining studies and different modeling methods, indicating robust results.

**Conclusions** This meta-analysis suggests that the UGT1A1*28 allele represents a biomarker for an increased risk of hyperbilirubinemia in HIV-positive patients receiving ATV.

## Introduction

Atazanavir (ATV) is currently one of the most widely used protease inhibitors in the treatment of HIV infection. It displays several advantages over other protease inhibitors, such as a favorable lipid profile, once daily dosing, low capsule burden, and a relatively distinct resistance profile [1]. The most frequent adverse effect associated with ATV use is an elevation of bilirubin. ATV causes hyperbilirubinemia due to inhibition of the enzyme uridine diphosphate glucuronosyltransferase 1A1 (UGT1A1), which is involved in the bilirubin conjugation [2]. The risk of hyperbilirubinemia is dependent on ATV plasma concentrations as well as genetic factors influencing UGT1A1 function [3,4].

The article "Association between the UGT1A1*28 allele and hyperbilirubinemia in HIV-positive patients receiving atazanavir: a meta-analysis" was published in 2019. Journal: Biosci Rep.

UGT1A1 is involved in the glucuronidation of several commonly used drugs, including gemfibrozil, ezetimibe, simvastatin, atorvastatin, cerivastatin, ethinylestradiol, buprenorphine, ibuprofen and ketoprofen [5–14]. An outstanding example is the glucuronidation and disposition to the side effects of the anticancer drug irinotecan [15–17]. Regarding the pharmacogenetics of Gilbert’s syndrome and drug side effects, there are two examples with mechanisms that are likely to influence the future administration of drugs, and potentially the drug-licensing process as well: irinotecan, the SN-38 metabolite of which is a UGT substrate, and ATV, which is not a substrate for glucuronidation, but nevertheless conveys a significant risk of unwanted jaundice by means of UGT inhibition [18].

There is some clinical controversy over the relevance of ATV-associated hyperbilirubinemia; it is benign and reversible upon discontinuation of the drug. Thus, some believe a proactive test in an attempt to predict and prevent its occurrence may not be warranted because they consider this adverse effect is not clinically relevant [19], whereas others maintain that this effect can be distressing and stigmatizing to patients and lead to increased discontinuation rates, so a preemptive screening test would be useful [20]. Up to now, there is no meta-analysis investigating this association. Therefore, we performed a meta-analysis to evaluate the association between the UGT1A1*28 allele and the associated hyperbilirubinemia risk.

## Methods

### Identification of eligible studies

Two independent investigators (P.D. and A.W.) carried out a systematic search in PubMed, Embase and Web of Sciences databases, with the last search update on 20 February 2019. The following search terms were used: (‘UGT1A1’ OR ‘UGT1A1*28’) AND ‘ATV’ AND (‘unconjugated hyperbilirubinemia’ OR ‘hyperbilirubinemia’), without any limitation applied. The reference lists of retrieved studies and recent reviews were also manually searched for further relevant studies.

### Inclusion and exclusion criteria

Hyperbilirubinemia refers to the accumulation of bilirubin in the blood causing jaundice. The clinical manifestations of jaundice are the skin, sclera and mucous membranes appear yellow. Studies in this meta-analysis must meet the following inclusion criteria: (i) evaluation of the association between UGT1A1*28 and hyperbilirubinemia; (ii) case–control study or cohort study; (iii) studies focusing on humans; and (iv) detailed genotype data in HIV-positive patients. Exclusion criteria: (i) duplication of previous publications; (ii) comment, review and editorial; and (iii) study with no detailed genotype data. Study selection was achieved by two investigators independently according to the inclusion and exclusion criteria by screening the title, abstract and full text. Any dispute was solved by discussion.

The article "Association between the UGT1A1*28 allele and hyperbilirubinemia in HIV-positive patients receiving atazanavir: a meta-analysis" was published in 2019. Journal: Biosci Rep.

### Data extraction and quality assessment

The data of the eligible studies were extracted in duplicate by two investigators independently (P.D. and X.L.). The following contents were collected: PMID, first author name, year of publication, country of origin, the characteristics of cases and controls, ethnicity, total bilirubin levels, sample size, Hardy–Weinberg equilibrium, number of cases and controls, study type and Newcastle–Ottawa Scale (NOS). The two authors checked the extracted data and reached a consensus on all data. If a dissent existed, they would recheck the original data of the included studies and have a discussion to reach a consensus. The authors used a quality score, ranging from 0 to 9, with higher scores associated with better study quality. Two investigators scored the studies independently and solved disagreements through discussion using the NOS Scoring system [21].

### Statistics analysis

Our analysis was conducted using the Review Manager Software 5.3 (Cochrane Collaboration, Oxford, U.K.). A chi-square-based Q test was used to measure heterogeneity between studies. In addition, an *I^2^* statistic was calculated to quantitate the proportion of the total variation across studies due to heterogeneity [22]. Fixed-effects and random-effects models were selected to analyze the data. Random-effects models were used only when there was a considerable heterogeneity (*P*<0.1 or I^2^ > 50%) among the studies. The overall effects were calculated by a combined Z value, with *P*<0.05 indicating statistical significance.

Odds ratios (OR) and 95% confidence intervals (95%CI) were calculated to evaluate the strength of the association between the UGT1A1*28 allele and its susceptibility to hyperbilirubinemia. The UGT1A1*28 allele contained UGT1A1 *1/*28 and *28/*28, and the common genotype was UGT1A1*1/*1. For the present study, we used the following group: (i) UGT1A1*28/*28 versus UGT1A1*1/*28; (ii) UGT1A1*1/*28 versus UGT1A1*1/*1; (iii) UGT1A1*28/*28 versus UGT1A1*1/*1; (iv) UGT1A1*28/*28 versus UGT1A1(*1/*28 + *1/*1); and (v) UGT1A1(*1/*28 + *28/*28) versus UGT1A1*1/*1.

### Sensitivity analysis and publication bias

Sensitivity analysis was conducted by the removal of each study, one at a time, understanding the effect of exclusion of respective studies by calculating the pooled ORs of the remaining studies. Heterogeneity was measured using *I^2^* values. If *I^2^* > 50% or *P*<0.1, we considered the study to have a great degree of heterogeneity and used a random-effects model. Otherwise, a fixed-effects model would be more appropriate.

The article "Association between the UGT1A1*28 allele and hyperbilirubinemia in HIV-positive patients receiving atazanavir: a meta-analysis" was published in 2019. Journal: Biosci Rep.

In addition, the fail-safe number, with significance set at 0.05 (Nfs_0.05_) for each meta-analysis, was applied to assess the publication bias. As a rule of thumb, if the Nfs_0.05_ was higher, the authors of the meta-analysis could be more comfortable assuming that the sample of studies was not likely to be overwhelmed by a future influx of studies with no significant relationship [23]. Nfs_0.05_ was calculated according to the formula:

(1) $${\text{Nfs}}_{0.05}\;=\;{\left(\text{SZ}/1.64\right)}^{2}\;-\;\text{k}$$

where k represents the number of included studies, Z represents the Z value of the independent study, and SZ is the sum of Z values [24].

## Results

### Characteristics of studies

A total of 102 studies were acquired from PubMed and Embase databases (PubMed: 37, Embase: 35, Web of Science: 30). Eighty-eight articles were excluded, of which 43 were duplicate articles and 45 had no relation to this topic. The remaining 14 studies were full-text reviewed, and 8 studies were excluded. Among these excluded studies were one having no relation to hyperbilirubinemia [25,26], one letter [27], one short communication [28], one case report [29], one systematic review [30], and two studies with no detailed genotype data [4,31]. The literature selection process is shown in Figure 1. Finally, six eligible studies [20,32–36] that met the inclusion criteria were included in our meta-analysis. The characteristics of each study are shown in Supplementary Material S1.

**Figure 1:** Flow chart for study identification, inclusion, and exclusion criteria

### UGT1A1*28/*28 versus UGT1A1*1/*28

Relevant data for the comparison of the risk of hyperbilirubinemia between HIV-positive patients with a UGT1A1*28/*28 genotype and those with a UGT1A1*1/*28 genotype was available in four of the included trials [33–36]. Pooled data from all studies showed that the risk of toxicity was higher among patients with a UGT1A1*28/*28 genotype than among those with a UGT1A1*1/*28 genotype (OR = 3.69, 95%CI = 1.82–7.49; *P*=0.0003). Heterogeneity was not statistically significant across all studies (*I^2^* = 27%, *P*=0.25) (Figure 2A).

**Figure 2:** Forest plots demonstrating the association between UGT1A1 allele and hyperbilirubinemia (**A**) UGT1A1*28/*28 versus UGT1A1*1/*28; (**B**) UGT1A1*1/*28 versus UGT1A1*1/*1; (**C**) UGT1A1*28/*28 versus UGT1A1*1/*1; (**D**) UGT1A1*28/*28 versus UGT1A1( *1/*28 + *1/*1 ); and (**E**) UGT1A1(*1/*28 + *28/*28) versus UGT1A1*1/*1.

The article "Association between the UGT1A1*28 allele and hyperbilirubinemia in HIV-positive patients receiving atazanavir: a meta-analysis" was published in 2019. Journal: Biosci Rep.

### UGT1A1*1/*28 versus UGT1A1*1/*1

A random-effects model was used due to the heterogeneity of *I^2^* > 50%. Four included trials compared the risk of hyperbilirubinemia between HIV-positive patients with a UGT1A1*1/*28 genotype and those with a wild-type allele [33–36]. A high level of heterogeneity was detected among these trials (*I^2^* = 61%, *P*=0.05). Overall analyses suggested an increased risk of hyperbilirubinemia in HIV-positive patients with a UGT1A1*1/*28 genotype as compared with those with a wild-type allele (OR = 3.50, 95%CI = 1.35–9.08; *P*=0.01) (Figure 2B).

### UGT1A1*28/*28 versus UGT1A1*1/*1

Four included trials compared the risk of unconjugated hyperbilirubinemia between HIV-positive patients with a UGT1A1*28/*28 genotype and those with a wild-type genotype [33–36]. Overall analyses suggested an increased risk of hyperbilirubinemia in HIV-positive patients with a UGT1A1*28/*28 genotype as compared with those with a wild-type genotype (OR = 10.07, 95%CI = 4.39–23.10; *P*<0.00001). No statistical heterogeneity was detected across all studies (*I^2^* = 0, *P*=0.55) (Figure 2C).

### UGT1A1*28/*28 versus UGT1A1(*1/*28 + *1/*1)

Five included trials compared the risk of hyperbilirubinemia between HIV-positive patients with a UGT1A1*28/*28 genotype and those with a UGT1A1*1/*28 or UGT1A1*1/*1 genotype [20,33–36]. Overall, analyses suggested an increased risk of hyperbilirubinemia in HIV-positive patients with a UGT1A1*28/*28 genotype as compared with those with a UGT1A1*1/*28 or UGT1A1*1/*1 genotype (OR = 5.91, 95%CI = 3.30–10.58; *P*<0.00001). No statistical heterogeneity was detected across all studies (*I^2^* = 0, *P*=0.46) (Figure 2D).

### UGT1A1(*1/*28 + *28/*28) versus UGT1A1*1/*1

Five included trials compared the risk of hyperbilirubinemia between HIV-positive patients with a UGT1A1*28 allele and those with a wild-type allele [32–36]. Four trials included patients with the UGT1A1*28 allele and wild-type allele that received ATV, and one trial compared receiving ATV with not receiving ATV among patients with a UGT1A1*28 allele and a wild-type allele. Four analyses suggested an increased risk of hyperbilirubinemia in HIV-positive patients with the UGT1A1*28 allele as compared with those with a wild-type allele (OR = 4.34, 95%CI = 2.55–7.39; *P*<0.00001). Moderate heterogeneity was detected across all studies (*I^2^* = 40%, *P*=0.17); and five analyses combined subgroup also suggested an increased risk of hyperbilirubinemia in HIV-positive patients with UGT1A1*28 allele as compared with those with a wild-type allele (OR = 4.89, 95%CI = 2.94–8.14; *P*<0.00001). Large heterogeneity was detected across all studies (*I^2^* = 54%, *P*=0.07) (Figure 2E).

The article "Association between the UGT1A1*28 allele and hyperbilirubinemia in HIV-positive patients receiving atazanavir: a meta-analysis" was published in 2019. Journal: Biosci Rep.

### Sensitivity and publication bias

All of the pooled ORs were not significantly affected by the remaining studies and different modeling methods, indicating robust results (Table 1). Moreover, the statistical outcomes of Orwin’s fail-safe N test are as follows: (1) UGT1A1*28/*28 versus UGT1A1*1/*28: Nfs_0.05_ = 2.50; (2) UGT1A1*1/*28 versus UGT1A1*1/*1: Nfs_0.05_ = 11.97; (3) UGT1A1*28/*28 versus UGT1A1*1/*1: Nfs_0.05_ = 23.94; (4) UGT1A1 (*1/*28 + *28/*28) versus UGT1A1*1/*1: Nfs_0.05_ = 48.03; and (v) UGT1A1*28/*28 versus UGT1A1 (*1/*28 + *1/*1): Nfs_0.05_ = 31.09. Based on these comprehensive quantitative evaluations, we concluded that no obvious publication bias existed in the assessed research.

**Table 1:** Sensitivity analysis of association between UGT1A1 alleles and hyperbilirubinemia

UGT1A1*28/*28 versus UGT1A1*1/*28		UGT1A1*1/*28 versus UGT1A1*1/*1		UGT1A1*28/*28 versus UGT1A1*1/*1		UGT1A1*28/*28 versus UGT1A1(*1/*28 + *1/*1)		UGT1A1 (*1/*28 + *28/*28) versus UGT1A1*1/*1	
Study exclusion	*P*-value	Study exclusion	*P*-value	Study exclusion	*P*-value	Study exclusion	*P*-value	Study exclusion	*P*-value
22661571	0.0003	22661571	0.01	22661571	<0.00001	22661571	<0.00001	22661571	<0.00001
17058217	0.002	17058217	<0.00001	17058217	0.0002	17058217	<0.0001	17058217	<0.00001
20504240	0.0005	20504240	0.002	20504240	<0.00001	21288825	<0.00001	20504240	<0.00001
23148286	0.0004	23148286	0.0001	23148286	<0.00001	20504240	<0.00001	23148286	<0.00001
						23148286	<0.00001	16170755	<0.00001

## Discussion

To the best of our knowledge, this is the first meta-analysis examining the effect of UGT1A1*28 polymorphism on the risk of hyperbilirubinemia in HIV-positive patients receiving ATV. The unconjugated bilirubin level was calculated by subtracting the conjugated bilirubin level from the total bilirubin level. Hyperbilirubinemia severity was classified on the basis of the AIDS Clinical Trial Group guidelines [37] for total bilirubin levels as follows: grade 1 (mild), 23–32 μM (1.3–1.9 mg/dl); grade 2 (moderate), 33–53 μM (1.9–3.1 mg/dl); grade 3 (severe), 54–105 μM (3.1–6.1 mg/dl); and grade 4 (serious), >105 μM (>6.1 mg/dl). This article refers specifically to severe and serious hyperbilirubinemia which was defined as grades 3 and 4 hyperbilirubinemia, respectively. Rotger et al. [32] provided the analysis that ATV increased bilirubin levels by 0.87 mg/dl, and indinavir increased bilirubin levels by 0.46 mg/dl. Ritonavir, lopinavir, saquinavir and nelfinavir had no or minimal effect on bilirubin levels. Ferraris et al. [34] provided the analysis that ritonavir removal was associated with a significant decrease in total bilirubin levels from 4.09 mg/dl (IQR: 3.14–5.73 mg/dl) to 1.82 mg/dl (IQR: 1.53–2.33 mg/dl) (*P*=0.001) in the remaining 24 patients in the switch arm, 12 months after therapy simplification, leading to a significant reduction in the number of patients presenting ≥ grade 3 hyperbilirubinemia. That means the combination of ritonavir and ATV increased the plasma concentration of ATV, which resulted in a higher bilirubin level than ATV alone. Bioequivalence between cobicistat and ritonavir as a pharmacoenhancer of ATV was established. Cobicistat shows increased advantages over ritonavir, such as no activity against HIV, fewer drug–drug interactions and better solubility, which promotes coformulation strategies with less pill burden, better tolerability, and, potentially, higher life-long treatment adherence [38]. Lankisch et al. [36] clarified that ATV therapy did not lead to hepatic toxicity indicated by aminotransferase elevations but rather resulted in a significantly higher rate of hyperbilirubinemia. The primary finding of the present study is that HIV-positive patients carrying UGT1A1*28 allele(s) including UGT1A1*1/*28 and UGT1A1*28/*28 are at an increased risk of hyperbilirubinemia than those carrying the UGT1A1*1/*1 allele. A secondary finding is that the UGT1A1*28/*28 allele has an increased risk compared with UGT1A1*1/*28 in HIV-positive patients receiving ATV.

The article "Association between the UGT1A1*28 allele and hyperbilirubinemia in HIV-positive patients receiving atazanavir: a meta-analysis" was published in 2019. Journal: Biosci Rep.

It is important to note that four additional important articles were not included in this meta-analysis (one letter, one short communication and two articles). The letter [25] and the short communication [26] were excluded because both studies were published as abstracts and the data were not presented in detail, but these conclusions confirmed a direct correlation between ATV plasma level and bilirubinemia that was influenced by the presence of a homozygosis or heterozygosis UGT1A1-TA7 (seven thymine–adenine) allele, and also confirmed our results that there was a significant association between UGT1A1*28 allele(s) and hyperbilirubinemia. Two articles [29,30] provided incomplete data concerning the association between UGT1A1*28 mutation and incidence of hyperbilirubinemia. However, taking these results into consideration will not change the result of our meta-analysis. For example, Javelle et al. [29] provided the analysis that having at least one of seven alleles at UGT1A1 was independently associated with severe hyperbilirubinemia (OR, 2.96; 95%CI, 1.29–6.78; *P*=0.01). Culley et al. [30] confirmed the association of hyperbilirubinemia with the use of an ATV/r-containing regimen in individuals carrying the UGT1A1 polymorphism, highlighting also the fact that carriers of the polymorphism develop total bilirubin levels >5 mg/dl in the majority of cases when on ATV/r. The risk for bilirubin-related ATV discontinuation is substantial, Lubomirov et al. [20] found that first-year cumulative rates of treatment discontinuation about UGT1A1 alleles were 62.5% for homozygous, 23.8% for heterozygous and 14.6% for noncarrier individuals. And for the four centers prescribing ATV to more than ten individuals, there was a statistically significant correlation between discontinuation rates and frequency of UGT1A1*28 homozygocity.

The article "Association between the UGT1A1*28 allele and hyperbilirubinemia in HIV-positive patients receiving atazanavir: a meta-analysis" was published in 2019. Journal: Biosci Rep.

UGT1A1 is a major conjugating enzyme responsible for bilirubin homeostasis [39], and it is expressed in the liver and gastrointestinal tract. One of the main functions of UGT1A1 lies within the liver, where it is the sole enzyme responsible for the metabolism of bilirubin, the hydrophobic breakdown product of hemecatabolism [18,40]. In general, UGT1A enzymes have considerable overlap in substrate specificities [41], however, no other isozyme can substitute for the bilirubin glucuronidation activity of UGT1A1 [18]. Additionally, no effective alternative pathways exist for the detoxification and elimination of bilirubin, excluding that of photoisomeration, a relatively inefficient pathway as compared with UGT1A1 glucuronidation [42]. Its activity is essential in the metabolism of bilirubin [43]. To date, more than 100 variants have been reported in the *UGT1A1* gene [44]. Some have been associated either with a decrease (e.g. UGT1A1*28, UGT1A1*6) or with an increase (e.g. UGTA1*36) in UGT1A1 metabolic function. The most thoroughly studied variant of UGT1A1 is termed as UGT1A1*28 (rs8175347) and is associated with Gilbert’s syndrome. This variant corresponds to a TA7 dinucleotide repeat in the TATA box at the promoter region of the *UGT1A1* gene as opposed to six (TA6) that characterizes the wild-type allele (UGT1A1*1) [45]. The distribution of the UGT1A1*28 allele varies across the globe with a minor allelic frequency (MAF) of 26–31% in Caucasians, 42–56% in African-Americans and only 9–16% in Asian populations [45,46]. Gilbert’s syndrome is characterized by mild and intermittent elevations of bilirubin caused by homozygosity of the c.-53-52 (TA)6 > (TA)7 allele in UGT1A1 at rs8175347 (*28). The UGT1A1 *28 allele consists of TA7 tandem repeats in the promoter region of UGT1A1 where normally there are six (UGT1A1*1 allele). The *28 allele causes approximately 50% decrease in UGT1A1 protein expression. Similarly, the *37 ((TA)8) allele also decreases UGT1A1 transcriptional activity relative to *28, whereas the *36 ((TA)5) allele in UGT1A1 leads to increased transcriptional activity relative to *28 [47]. The *36 and *37 alleles are rare in White and Asian populations, but are more common in West and sub-Saharan African populations [48]. The UGT1A1*6 allele (c.211 G>A at rs4148323), which causes a missense mutation (G71R), is more prevalent in individuals of East Asian descent, but has not been found to be associated with ATV-associated hyperbilirubinemia [35].

The article "Association between the UGT1A1*28 allele and hyperbilirubinemia in HIV-positive patients receiving atazanavir: a meta-analysis" was published in 2019. Journal: Biosci Rep.

Polymorphisms in UGT1A1 are associated with indirect bilirubin concentrations in the general population (i.e. Gilbert’s syndrome). Polymorphisms in genes beyond UGT1A1 have been reported to be associated with serum bilirubin concentrations in the general population, including ABCC2, ABCB4, ABCB11, ATP8B1, SLCO1B1 [49], SLCO1B3 and G6PD [50]. In addition, bilirubin concentrations have been associated with ABCB1 3435C>T among patients prescribed ATV without ritonavir but not with ritonavir alone [26], although results have been inconsistent [4].

Limitations of this meta-analysis must be considered. First, the possibility of information and selection biases cannot be completely excluded because some of the included studies were retrospective. Second, we restricted our search to articles published in English or Chinese. Articles with potentially high-quality data that were published in other languages were not included because of anticipated difficulties in obtaining accurate medical translation. Third, our study did not make the correlation analysis of ethnicity and drug doses. Finally, the association of hyperbilirubinemia and ATV mainly occurs when ATV is boosted. Hypothetical selection bias could have selected patients all with boosted ATV, and that this association might not exist in non-boosted ATV regimens.

In conclusion, the presence of the UGT1A1*28 allele with ATV use increases the risk of developing severe hyperbilirubinemia. Although hyperbilirubinemia is considered a mild adverse effect, it has clinical implications. Jaundice causes discomfort due to the yellowish appearance of the skin, which may affect the quality of life of these patients and may lead to treatment discontinuation. It is important to keep in mind that the variant allele frequencies should be considered in each population before initiating a genotyping program.

## Supporting information

**Supplementary Material S1:** 

## Abbreviations

ATV: atazanavir
95%CI: 95% confidence interval
NOS: Newcastle–Ottawa Scale
OR: odds ratio
TA7: seven thymine–adenine
UGT1A1: uridine diphosphate glucuronosyltransferase 1A1

The article "Association between the UGT1A1*28 allele and hyperbilirubinemia in HIV-positive patients receiving atazanavir: a meta-analysis" was published in 2019. Journal: Biosci Rep.

## References

[1] RivasP., MorelloJ., GarridoC., Rodriguez-NovoaS. and SorianoV. (2009) Role of atazanavir in the treatment of HIV infection. Ther. Clin. Risk Manag. 5, 99–116 19436623PMC2697529

[2] ZhangD., ChandoT.J., EverettD.W., PattenC.J., DehalS.S. and HumphreysW.G. (2005) In vitro inhibition of UDP glucuronosyltransferases by atazanavir and other HIV protease inhibitors and the relationship of this property to in vivo bilirubin glucuronidation. Drug Metab. Dispos. 33, 1729–1739 10.1124/dmd.105.005447 16118329

[3] Rodriguez NovoaS., BarreiroP., RendonA., BarriosA., CorralA., Jimenez-NacherI. (2006) Plasma levels of atazanavir and the risk of hyperbilirubinemia are predicted by the 3435C–>T polymorphism at the multidrug resistance gene 1. Clin. Infect. Dis. 42, 291–295 1635534410.1086/499056

[4] Rodriguez-NovoaS., Martin-CarboneroL., BarreiroP., Gonzalez-PardoG., Jimenez-NacherI., Gonzalez-LahozJ. (2007) Genetic factors influencing atazanavir plasma concentrations and the risk of severe hyperbilirubinemia. AIDS 21, 41–46 10.1097/QAD.0b013e328011d7c1 17148966

[5] SparksR., UlrichC.M., BiglerJ., TworogerS.S., YasuiY., RajanK.B. (2004) UDP-glucuronosyltransferase and sulfotransferase polymorphisms, sex hormone concentrations, and tumor receptor status in breast cancer patients. Breast Cancer Res. 6, R488–R498 10.1186/bcr818 15318931PMC549165

[6] AdegokeO.J., ShuX.O., GaoY.T., CaiQ., BreyerJ., SmithJ. (2004) Genetic polymorphisms in uridine diphospho-glucuronosyltransferase 1A1 (UGT1A1) and risk of breast cancer. Breast Cancer Res. Treat. 85, 239–245 10.1023/B:BREA.0000025419.26423.b8 15111762

[7] CecchinE., RussoA., CoronaG., CampagnuttaE., MartellaL., BoiocchiM. (2004) UGT1A1*28 polymorphism in ovarian cancer patients. Oncol. Rep. 12, 457–462 15254716

[8] ChouinardS., TessierM., VernouilletG., GauthierS., LabrieF., BarbierO. (2006) Inactivation of the pure antiestrogen fulvestrant and other synthetic estrogen molecules by UDP-glucuronosyltransferase 1A enzymes expressed in breast tissue. Mol. Pharmacol. 69, 908–920 1633938910.1124/mol.105.015891

[9] EbnerT., RemmelR.P. and BurchellB. (1993) Human bilirubin UDP-glucuronosyltransferase catalyzes the glucuronidation of ethinylestradiol. Mol. Pharmacol. 43, 649–654 8474433

[10] GhosalA., HapangamaN., YuanY., Achanfuo-YeboahJ., IannucciR., ChowdhuryS. (2004) Identification of human UDP-glucuronosyltransferase enzyme(s) responsible for the glucuronidation of ezetimibe (Zetia). Drug Metab. Dispos. 32, 314–320 10.1124/dmd.32.3.314 14977865

[11] KingC.D., RiosG.R., GreenM.D., MacKenzieP.I. and TephlyT.R. (1997) Comparison of stably expressed rat UGT1.1 and UGT2B1 in the glucuronidation of opioid compounds. Drug Metab. Dispos. 25, 251–255 9029056

The article "Association between the UGT1A1*28 allele and hyperbilirubinemia in HIV-positive patients receiving atazanavir: a meta-analysis" was published in 2019. Journal: Biosci Rep.

[12] KuehlG.E., LampeJ.W., PotterJ.D. and BiglerJ. (2005) Glucuronidation of nonsteroidal anti-inflammatory drugs: identifying the enzymes responsible in human liver microsomes. Drug Metab. Dispos. 33, 1027–1035 10.1124/dmd.104.002527 15843492

[13] OgilvieB.W., ZhangD., LiW., RodriguesA.D., GipsonA.E., HolsappleJ. (2006) Glucuronidation converts gemfibrozil to a potent, metabolism-dependent inhibitor of CYP2C8: implications for drug-drug interactions. Drug Metab. Dispos. 34, 191–197 10.1124/dmd.105.007633 16299161

[14] PrueksaritanontT., SubramanianR., FangX., MaB., QiuY., LinJ.H. (2002) Glucuronidation of statins in animals and humans: a novel mechanism of statin lactonization. Drug Metab. Dispos. 30, 505–512 10.1124/dmd.30.5.505 11950779

[15] LankischT.O., VogelA., EilermannS., FiebelerA., KroneB., BarutA. (2005) Identification and characterization of a functional TATA box polymorphism of the UDP glucuronosyltransferase 1A7 gene. Mol. Pharmacol. 67, 1732–1739 10.1124/mol.104.007146 15716465

[16] InnocentiF., VokesE.E. and RatainM.J. (2006) Irinogenetics: what is the right star? J. Clin. Oncol. 24, 2221–2224 10.1200/JCO.2005.05.2464 16636339

[17] AndoY., SakaH., AsaiG., SugiuraS., ShimokataK. and KamatakiT. (1998) UGT1A1 genotypes and glucuronidation of SN-38, the active metabolite of irinotecan. Ann. Oncol. 9, 845–847 10.1023/A:1008438109725 9789606

[18] StrassburgC.P. (2008) Pharmacogenetics of Gilbert’s syndrome. Pharmacogenomics 9, 703–715 10.2217/14622416.9.6.703 18518849

[19] NettlesR.E., ChildM.J., BertzR.J. and SchnittmanS. (2006) Gilbert syndrome and the development of antiretroviral therapy-associated hyperbilirubinemia: genetic screening is unnecessary. J. Infect. Dis. 193, 1611–1612, 10.1086/503814 16652295

[20] LubomirovR., ColomboS., di IulioJ., LedergerberB., MartinezR., CavassiniM. (2011) Association of pharmacogenetic markers with premature discontinuation of first-line anti-HIV therapy: an observational cohort study. J. Infect. Dis. 203, 246–257 10.1093/infdis/jiq043 21288825PMC3071070

[21] LoC.K., MertzD. and LoebM. (2014) Newcastle-Ottawa Scale: comparing reviewers’ to authors’ assessments. BMC Med. Res. Methodol. 14, 45 10.1186/1471-2288-14-45 24690082PMC4021422

[22] HigginsJ.P., ThompsonS.G., DeeksJ.J. and AltmanD.G. (2003) Measuring inconsistency in meta-analyses. BMJ 327, 557–560 10.1136/bmj.327.7414.557 12958120PMC192859

[23] LiX., YuK., MeiS., HuoJ., WangJ., ZhuY. (2015) HLA-B*1502 increases the risk of phenytoin or lamotrigine induced Stevens-Johnson Syndrome/toxic epidermal necrolysis: evidence from a meta-analysis of nine case-control studies. Drug Res. 65, 107–111 2487193110.1055/s-0034-1375684

The article "Association between the UGT1A1*28 allele and hyperbilirubinemia in HIV-positive patients receiving atazanavir: a meta-analysis" was published in 2019. Journal: Biosci Rep.

[24] ShenS.D., ZhongS.Z., WangC.Z. and HuangW.H. (2015) Correlation of lymphovascular invasion with clinicopathological factors in invasive breast cancer: a meta-analysis. Int. J. Clin. Exp. Med. 8, 17789–17795 26770370PMC4694270

[25] TsaiM.S., ChangS.Y., LinS.W., KuoC.H., SunH.Y., WuB.R. (2017) Treatment response to unboosted atazanavir in combination with tenofovir disoproxil fumarate and lamivudine in human immunodeficiency virus-1-infected patients who have achieved virological suppression: A therapeutic drug monitoring and pharmacogenetic study. J. Microbiol. Immunol. Infect. 50, 789–797 10.1016/j.jmii.2015.12.012 26857335

[26] AndersonP.L., AquilanteC.L., GardnerE.M., PredhommeJ., McDaneldP., BushmanL.R. (2009) Atazanavir pharmacokinetics in genetically determined CYP3A5 expressors versus non-expressors. J. Antimicrob. Chemother. 64, 1071–1079 10.1093/jac/dkp317 19710077PMC2760462

[27] CicconiP., BiniT., BarassiA., CasanaM., TurriO., PateriF. (2011) Detrimental effect of atazanavir plasma concentrations on total serum bilirubin levels in the presence of UGT1A1 polymorphisms. J. Acquir. Immune Defic. Syndr. 56, e96–97 10.1097/QAI.0b013e318203e7e7 21317582

[28] MorelloJ., AlvarezE., CuencaL., VispoE., Gonzalez-LahozJ., SorianoV. (2011) Short communication: use of serum bilirubin levels as surrogate marker of early virological response to atazanavir-based antiretroviral therapy. AIDS Res. Hum. Retroviruses 27, 1043–1045 10.1089/aid.2011.0019 21348813

[29] JavelleE., OliverM., SaviniH., AubryC., BadensC. and SimonF. (2012) Severe atazanavir-associated hyperbilirubinemia revealing Canton G6PD deficiency in an Asian HIV-infected patient. AIDS 26, 249–251 10.1097/QAD.0b013e32834e1d33 22179231

[30] CulleyC.L., KiangT.K., GilchristS.E. and EnsomM.H. (2013) Effect of the UGT1A1*28 allele on unconjugated hyperbilirubinemia in HIV-positive patients receiving Atazanavir: a systematic review. Ann. Pharmacother. 47, 561–572 10.1345/aph.1R550 23548653

[31] PanagopoulosP., ParaskevisD., KatsarolisI., SypsaV., DetsikaM., ProtopapasK. (2014) High prevalence of the UGT1A1*28 variant in HIV-infected individuals in Greece. Int. J. STD AIDS 25, 860–865 10.1177/0956462414523259 24516079

[32] RotgerM., TaffeP., BleiberG., GunthardH.F., FurrerH., VernazzaP. (2005) Gilbert syndrome and the development of antiretroviral therapy-associated hyperbilirubinemia. J. Infect. Dis. 192, 1381–1386 10.1086/466531 16170755

[33] RibaudoH.J., DaarE.S., TierneyC., MorseG.D., MollanK., SaxP.E. (2013) Impact of UGT1A1 Gilbert variant on discontinuation of ritonavir-boosted atazanavir in AIDS Clinical Trials Group Study A5202. J. Infect. Dis. 207, 420–425 10.1093/infdis/jis690 23148286PMC3537445

The article "Association between the UGT1A1*28 allele and hyperbilirubinemia in HIV-positive patients receiving atazanavir: a meta-analysis" was published in 2019. Journal: Biosci Rep.

[34] FerrarisL., ViganoO., PeriA., TarkowskiM., MilaniG., BonoraS. (2012) Switching to unboosted atazanavir reduces bilirubin and triglycerides without compromising treatment efficacy in UGT1A1*28 polymorphism carriers. J. Antimicrob. Chemother. 67, 2236–2242 10.1093/jac/dks175 22661571

[35] ParkW.B., ChoeP.G., SongK.H., JeonJ.H., ParkS.W., KimH.B. (2010) Genetic factors influencing severe atazanavir-associated hyperbilirubinemia in a population with low UDP-glucuronosyltransferase 1A1*28 allele frequency. Clin. Infect. Dis. 51, 101–106 10.1086/653427 20504240

[36] LankischT.O., MoebiusU., WehmeierM., BehrensG., MannsM.P., SchmidtR.E. (2006) Gilbert’s disease and atazanavir: from phenotype to UDP-glucuronosyltransferase haplotype. Hepatology 44, 1324–1332 10.1002/hep.21361 17058217

[37] FellayJ., BoubakerK., LedergerberB., BernasconiE., FurrerH., BattegayM. (2001) Prevalence of adverse events associated with potent antiretroviral treatment: Swiss HIV Cohort Study. Lancet 358, 1322–1327 10.1016/S0140-6736(01)06413-3 11684213

[38] AntunesF. (2017) Atazanavir sulfate + cobicistat for the treatment of HIV infection. Expert Rev. Anti Infect. Ther. 15, 569–576 10.1080/14787210.2017.1323634 28443391

[39] KiangT.K., EnsomM.H. and ChangT.K. (2005) UDP-glucuronosyltransferases and clinical drug-drug interactions. Pharmacol. Ther. 106, 97–132 10.1016/j.pharmthera.2004.10.013 15781124

[40] BosmaP.J., SeppenJ., GoldhoornB., BakkerC., Oude ElferinkR.P., ChowdhuryJ.R. (1994) Bilirubin UDP-glucuronosyltransferase 1 is the only relevant bilirubin glucuronidating isoform in man. J. Biol. Chem. 269, 17960–17964 8027054

[41] TukeyR.H. and StrassburgC.P. (2000) Human UDP-glucuronosyltransferases: metabolism, expression, and disease. Annu. Rev. Pharmacol. Toxicol. 40, 581–616 10.1146/annurev.pharmtox.40.1.581 10836148

[42] SchauerR., StanglM., LangT., ZimmermannA., ChoukerA., GerbesA.L. (2003) Treatment of Crigler-Najjar type 1 disease: relevance of early liver transplantation. J. Pediatr. Surg. 38, 1227–1231 10.1016/S0022-3468(03)00273-2 12891498

[43] Radominska-PandyaA., CzernikP.J., LittleJ.M., BattagliaE. and MackenzieP.I. (1999) Structural and functional studies of UDP-glucuronosyltransferases. Drug Metab. Rev. 31, 817–899 10.1081/DMR-100101944 10575553

[44] MarquesS.C. and IkediobiO.N. (2010) The clinical application of UGT1A1 pharmacogenetic testing: gene-environment interactions. Hum. Genomics 4, 238–249 2051113710.1186/1479-7364-4-4-238PMC3525209

[45] BosmaP.J., ChowdhuryJ.R., BakkerC., GantlaS., de BoerA., OostraB.A. (1995) The genetic basis of the reduced expression of bilirubin UDP-glucuronosyltransferase 1 in Gilbert’s syndrome. N. Engl. J. Med. 333, 1171–1175 10.1056/NEJM199511023331802 7565971

The article "Association between the UGT1A1*28 allele and hyperbilirubinemia in HIV-positive patients receiving atazanavir: a meta-analysis" was published in 2019. Journal: Biosci Rep.

[46] BeutlerE., GelbartT. and DeminaA. (1998) Racial variability in the UDP-glucuronosyltransferase 1 (UGT1A1) promoter: a balanced polymorphism for regulation of bilirubin metabolism? Proc. Natl. Acad. Sci. U.S.A. 95, 8170–8174 10.1073/pnas.95.14.8170 9653159PMC20948

[47] MemonN., WeinbergerB.I., HegyiT. and AleksunesL.M. (2016) Inherited disorders of bilirubin clearance. Pediatr. Res. 79, 378–386 10.1038/pr.2015.247 26595536PMC4821713

[48] HorsfallL.J., ZeitlynD., TarekegnA., BekeleE., ThomasM.G., BradmanN. (2011) Prevalence of clinically relevant UGT1A alleles and haplotypes in African populations. Ann. Hum. Genet. 75, 236–246 10.1111/j.1469-1809.2010.00638.x 21309756

[49] SannaS., BusoneroF., MaschioA., McArdleP.F., UsalaG., DeiM. (2009) Common variants in the SLCO1B3 locus are associated with bilirubin levels and unconjugated hyperbilirubinemia. Hum. Mol. Genet. 18, 2711–2718 10.1093/hmg/ddp203 19419973PMC2701337

[50] JohnsonA.D., KavousiM., SmithA.V., ChenM.H., DehghanA., AspelundT. (2009) Genome-wide association meta-analysis for total serum bilirubin levels. Hum. Mol. Genet. 18, 2700–2710 10.1093/hmg/ddp202 19414484PMC2701336

